RETRACTED

# Role of Human-Computer Interaction Healthcare System in the Teaching of Physiology and Medicine

**DOI:** 10.1155/2022/5849736

**Published:** 2022-04-13

**Authors:** Xiuhong Li, Yubo Xu

**Affiliations:** ^1^Linfen Vocational and Technical College, Linfen 041000, Shanxi, China; ^2^School of Information Science and Technology, Xiamen University Tan Kah Kee College, Zhangzhou 363000, Fujian, China

## Abstract

With the increasingly severe aging of the population, the difficult and expensive medical treatment problems are becoming more and more prominent; the salary level of domestic doctors is not high, but the cost of training doctors is high, coupled with doctors' work pressure and mental pressure; the number of candidates for medical school is decreasing year by year; medical talent is rare; and the allocation of medical staff is scarce. Health care is the basic guarantee for people's good life, and the shortage of medical staff will have many impacts on health care. Human-computer interaction (HCI) is the study of people, computers, and their interaction. HCI refers to the communication between the user and the computer system, which is the two-way information exchange of various symbols and actions between the human and the computer. The purpose of this paper is to study a healthcare system with human-computer interaction through the client, apply the system to the teaching of physiology and medicine, and analyze its effects and functions in combination with various evaluation indicators. This paper selects teaching content, ease of use of human-computer interaction design, technical services, and user subjective satisfaction as evaluation indicators, and constructs an evaluation model for this. And it builds the physiology and medicine teaching system framework and healthcare system, and conducts tests and statistics on the teaching system. This paper combines online questionnaires, in-app survey feedback, and field visits to collect feedback from users and administrators. The final data show that the teaching system meets the requirements in four evaluation indicators: teaching content, ease of use of human-computer interaction design, technical services, and user subjective satisfaction. User satisfaction with these four aspects reached 86.33%, 95.17%, 63.83%, and 81.87%, respectively. It shows that the system is more popular and can meet the needs of most users.

## 1. Introduction

The interaction between humans and computers is created by the development of industrial design. It is the link for people to use machines for daily life and production activities, and it is a necessary process for people to “communicate” with machines. Since the advent of computers, almost all human life has been closely linked to information technology, and the way people continue to interact smoothly with computers is the computer interface. Today, the design is focused on user experience and quality of life almost everywhere. Correspondingly, the design of human-computer interaction interface affects the user's operation mode and device experience, and plays a crucial role in the practicability and ease of use of machines and computer equipment.

RETRACTED

In the medical and health field, human-machine interface design is more specific and rigorous. Due to its monitoring and reference functions, medical monitoring equipment requires more accurate and accurate expression, and timely and simple operation. Therefore, the human-computer interaction design of the medical monitoring equipment interface is particularly important. As far as the domestic situation is concerned, with the awakening and development of design consciousness, people gradually begin to pay attention to the application of design aesthetics in production and life, including health and medical equipment.

At present, foreign medical device design is mainly based on graphic interface, while domestic design is mainly based on catching up with foreign technology and modeling design. At the same time, the home medical equipment does not consider the human-computer interaction of the user interface, resulting in confusion in the identification of the user interface and passive operation of the user. Therefore, when it comes to the user interface of domestic medical devices, it is necessary to emphasize the design concept of comfort and humanization, which is also the basic way to create a harmonious interaction between users and products.

Markets and hospitals have medical device models from different national brands. Although the functions are similar, the operation methods are different, so the learning cost is high and the error rate is high. High-end medical devices are related to the safety of people, and the design of human-computer interaction needs to be carefully considered in the research and development of medical devices. In the development of medical devices, the design of human-computer interaction needs to be carefully considered. In the development of medical devices, the design of human-computer interaction needs to be carefully considered. Make it adapt to people's use habits and the characteristics of enabling material, color, and touch, and reduce the fault tolerance rate of medical staff.

## 2. Related Work

With the development of society and the improvement of people's living standards, people's requirements for health care are getting higher and higher. At present, many scholars have carried out related research on this. Hynes SO suggested that a unified integrative approach could be employed to address multiple driver mutations, using next-generation sequencing (NGS) combined with morpho-molecular approaches to treat tumors. There are still challenges in applying NGS to routine clinical practice, which include validation, processing large streams of information, and generating clinically useful reports. These challenges are particularly acute in UHC (Universal Healthcare) settings. These challenges are particularly acute in the UHC (Universal Healthcare) setting, as the UHC is unable to repay the testing costs and has limited available resources. Hynes SO believes that the challenges of applying NGS in the UHC environment are surmountable. Hynes S O outlines its routine application in diagnostics, clinical trials, and research paradigms [1]. To prevent lifestyle diseases, wearable biosignal monitoring systems for daily monitoring have attracted attention. Izumi S introduced electrocardiograph (ECG) processors used in wearable medical systems. It includes an analog front-end, a 12-bit ADC, a powerful instantaneous heart rate (IHR) monitor, a 32-bit Cortex-M0 kernel, and a 64-KB ferroelectric random access memory (FeRAM). Although IHR (Instantaneous Heart Rate) monitors are used in noisy conditions, a short-term autocorrelation (STAC) algorithm is used to improve the accuracy of heart rate detection [2]. In the face of fragmented and underperforming healthcare delivery systems, Gonzalo J D examines the current state of medical education in relation to system science and proposes a new framework for educating physicians to adapt and practice systems-based environments. Specifically, Gonzalo J D proposes a shift in education from a two-pillar framework to a three-pillar framework in which basic, clinical, and system sciences are interdependent. In this new three-pillar framework, students not only learn the interconnections between basic, clinical, and system sciences, but also reveal relevance and meaning care systems in their education through their authentic, value-added, and patient-centered role as pilots in the health field. Gonzalo J D describes the systems navigation course currently implemented for all students at Penn State School of Medicine. As an example of this three-pillar educational model, adequate preparation requires a clear focus on systems science as an important and equal component of physician education [3]. Gesture recognition is crucial in the field of human-computer interaction, especially in health care, rehabilitation, sign language translation, and more. Traditionally, gesture recognition data collected by the inertial measurement unit (IMU) sensors are forwarded to the cloud or to remote devices with higher computing power to train the model. However, remote tracking therapy for exercise rehabilitation training is not convenient, and Jiang W proposes a wearable deep learning system capable of processing data locally on end devices based on a field programmable gate array (FPGA) accelerator and a Cortex-M0 IP core. The device uses a preprocessing module and a string mix, with low power consumption and low latency at the microcontrol unit (MCU) level, but achieves or exceeds the performance of a single-board computer (SBC). Furthermore, Convolutional Neural Network (CNN) and Multilayer Perceptron Neural Network (NN) are used in the recognition model to extract features and classify gestures, which helps achieve a recognition accuracy of up to 97%. Finally, Jiang W provides a software-hardware co-design method, which is worthy of reference for the design of edge devices in other scenarios [4]. With the rise of robotic surgical systems, medical patients using AI human-computer interaction technology and now requirements around electronic health records (EHR) are examine these systems as part of their larger sociotechnical systems. As human-computer interaction (HCI) research in healthcare settings continues to increase, Vo V H examines this phenomenon based on a previous trend analysis published as a HFES program from 1999 to 2009 for a specific domain of HCI healthcare. Vo V H explores trends in healthcare procedures published by HFES from 2009 to 2017, discussing changes in trends and their implications [5]. In recent years, recognizing human activities in everyday environments has attracted a lot of research in computer vision and recognition. In addition, it is also very valuable for many practical applications such as smart home, gaming, health care, human-computer interaction, and robotics, where intelligent systems are now the most important topic. In this study, Li Z proposes a new method for everyday activity recognition and hypothesizes that the performance of the system can be improved by incorporating multimodal features. Li Z extracted the spatiotemporal features of human body based on the bone data in RGB-D data and represented with parts. Li Z then combines multiple features from both sources to produce robust features for activity representation. Finally, Li Z uses a multicore learning algorithm to fuse multiple features to identify active labels for each video. To show generality, the proposed framework has been tested on two challenging datasets through a cross-validation scheme. The experimental results show good results on both CAD120 and MSR-Daily Activity 3D datasets, with accuracy rates of 94.16% and 95.31%, respectively [6]. Mohan, P performed a series of simulations to ensure the performance improvement of IMCMR-UWSN technology, the comparative results demonstrate the superiority of IMCMR-UWSN technology in terms of different measures. Rawat S.S mathematically solves the proposed TV-PSMSV method using an alternating direction multiplier (ADMM) to validate the proposed solution. Experimental evaluation using real and synthetic datasets shows that the proposed TV-PSMSV outperforms existing reference methods in background repressor (BSF) and letter gain ratio (SCRG). Mani V proposed an innovative solution, patient-centered healthcare data management (PCHDM), regarding distributed ledger technology performance. Mani, V tested against superledger calipers in terms of transaction delays, resource utilization, and transaction volume per second. The results show that the model gives stakeholders more confidence in collaborating and sharing their health records.

RETRACTED

## 3. Healthcare System Based on Human-Computer Interaction

### 3.1. Healthcare System

1. Current status of health care. Health care is the guarantee of a better life for the people. As a country with a large population in the world, China has a huge demand for medical services and stricter requirements for the construction of a healthcare system. This paper sorts out the domestic healthcare demand market and the application market of medical devices in recent years; according to the relevant public information, this paper has sorted out the domestic health and medical demand market and the application market conditions of medical devices in recent years, as shown in Figure 1 [7].
2. As can be seen from Figure 1(a), the use of medical rehabilitation equipment has increased in recent years. Among them, the use of magnetic stimulation rehabilitation medical equipment is increasing, and it is currently the most widely used. The second is electrical stimulation rehabilitation medical equipment, and the use of medical robots is gradually increasing. According to this trend, it is likely to exceed electrical stimulation rehabilitation medical equipment. In Figure 1(b), we can also see that the market size of domestic health examinations continues to increase, exceeding 190 billion yuan by 2020, which also reflects that people are paying more and more attention to their own health [8].
3. Problems faced by domestic health care. China's society and economy are still in a stage of rapid change and rapid development, the allocation of social resources has not yet reached the optimal allocation, and there are still some contradictions in the field of health care, which is fundamental to people's livelihood. For example, medical resources are not sufficient, the distribution of resources is uneven, and the medical system is not perfect.  Table 1 shows the development of domestic health and medical institutions according to relevant statistics [9].

RETRACTED

It can be seen from Table 1 that there are only 8.84 million domestic health technicians. Compared with the national population, there are only about 2 professional doctors per thousand people, while developed countries such as Switzerland and France have about four professional doctors per thousand people, which show that domestic medical resources are not sufficient. In addition to the lack of overall resources, domestic medical resources are not evenly distributed. On the basis of the relatively thin domestic medical resources, the uneven distribution of resources has exacerbated the shortage of medical resources in some remote areas [10, 11].

Figure 2 shows the traditional medical system. Traditional medical treatment involves several processes, such as appointment registration, queuing for medical treatment, symptomatic treatment, and review. This medical treatment method is inefficient, time-consuming, and labor-intensive, and the diagnosis method is single; the process is cumbersome.

### 3.2. Teaching of Physiology and Medicine

1. The current situation of physiology and medicine teaching. In order to fill the huge gap of domestic healthcare technicians and improve people's healthcare knowledge, it is necessary to carry out various aspects of physiology and medicine teaching. Traditional physiology and medicine teaching courses are limited to specialized places such as schools and hospitals, and the teaching objects are generally the groups of teachers and students related to majors, as shown in Figure 3. Everyone knows that health care is related to everyone, and everyone should be able to learn healthcare knowledge anytime, anywhere, regardless of age, so as to better promote national health care. With the development of the Internet and the innovation of the domestic education system, online education has been widely promoted and used. Network education has many advantages, such as learning anytime, anywhere, low teaching cost, diversified teaching courses, and retrospective teaching content, which can just solve the problems faced by physiology and medicine teaching [12, 13].
2. Physiological and medical teaching combined with the Internet. Medical education is not just about teaching traditional medical knowledge and theories, and the development of modern medicine requires medical educators to keep up with the development of medicine. Medical educators can access the latest data online and post their information, opinions, and achievements on relevant websites. In addition, in medical education, it is often difficult to directly display educational content such as human body structure, disease occurrence, and progress, and it is not easy to display various organisms and operations for a long time. However, through the CAI demonstration, better, more intuitive, and longer education quality and effects can be achieved [14, 15].

RETRACTED

### 3.3. Human-Computer Interaction

1. Concept. Among the tasks performed by computers, many tasks are performed by human-machine cooperation. In this case, humans and computers need to communicate with each other, which is called human-computer interaction, as shown in Figure 4.
2. Origin and development. It is generally divided into four stages: from the concept of “close human-machine coexistence” proposed in 1960 as the enlightenment point of view of human-machine interaction to the stage of the International Conference on Human-Machine Systems in 1969 as the founding period; from 1970 to 1979, many monographs were published and two research centers were established as the foundation period; from 1980 to 1995, many monographs were published successively, together with the latest research results and the improvement of the theoretical system, as the development period; since 1996, with the continuous maturity of computer technology and artificial intelligence, human-computer interaction is gradually approaching the maturity of “human-centered” [16, 17].
3. Human-computer interaction design. The elements required for human-computer interaction design are people, actions that people issue commands, and machines, also known as human factors, activity factors, and object factors. The goal of human-computer interaction design is to realize the user's mental model, so as to complete the user's goal. In the process of realizing the user's mental model, attention should be paid to the usability, dynamism, ease of use, diversity, and pleasure of human-computer interaction design. There is a big difference between traditional interaction design principles and modern interaction design principles, which can be seen from Figure 5 [18].
4. Classification of human-computer interaction. Human-machine interface can be divided into functional human-machine interface, emotional human-machine interface, and environmental human-machine interface. These three categories are not independent of each other, but have complex connections between them. Functional human-computer interface, namely, functional information on human-computer interaction objects, controls, and control objects, and also includes the docking with the manufacturing process, namely, the application of materials and technologies. Functional interface reflects the coordination between design and artificial objects; emotional human-machine interface, namely, objects need to convey emotions through the interface, and return to people, and have emotional resonance with people. The transmission of this kind of perceptual information has both predetermined information and differences between person and conditions, which is the unity of established content and unknown emotions. Environmental human-machine interface is the communication between external environmental factors and human beings. Products are inseparable from the environment, and the physical conditions and spiritual atmosphere of the environment are essential interface elements [19, 20].
5. Healthcare system based on human-computer interaction. At present, the domestic healthcare system mainly includes medical security system, medical facility management system, medical institution service system, medicine management system, and medical teaching system, as shown in Figure 6 [21]. The medical teaching system mainly includes the teaching of sports medicine, psychological medicine, psychiatry, diving medicine, aerospace medicine, navigation medicine, ultrasound medicine, biomedical engineering, forensic medicine, emergency medicine, epidemiology, social medicine, medical ethics, medicine overview, and so on.

RETRACTED

## 4. Performance Test of Healthcare System Based on HCI

### 4.1. HCI-Based Medical Teaching System

(1) Teaching system evaluation model. The evaluation indicators include teaching content, ease of use of human-computer interaction design, technical services, and user subjective satisfaction, as shown in Table 2.
The initial weight coefficient Wi' can be calculated by the geometric mean method
  (1) $$\begin{array}{c} W_{i}^{\prime }=\sqrt[{m}]{a_{i1}a_{i2}\cdots a_{\text{im}}}. \end{array}$$
In the formula, *m* is the number of subobjectives, and the normalized weight coefficient is obtained as follows:
  (2) $$\begin{array}{c} W_{i}=\frac{W_{i}^{\prime }}{\sum_{i=1}^{m}W_{i}^{\prime }}. \end{array}$$
Combined with AHP and checking the rationality of the coefficients, we can get
  (3) $$\begin{array}{c} \text{CI}=\frac{\lambda_{\max}-m}{m-1}. \end{array}$$
Among them, when CI < 0.1 is logically reasonable, *λ*_max_ is the largest eigenvalue, and
  (4) $$\begin{array}{c} \lambda_{\max}=\sum_{i=1}^{m}\frac{\lambda_{i}}{m},\\ \lambda_{i}=\sum_{j=1}^{m}\frac{a_{\text{ij}}w_{j}}{w_{i}}. \end{array}$$
Using RI to represent the average random consistency ratio, then the random consistency ratio CR is as follows:
  (5) $$\begin{array}{c} \text{CR}=\frac{\text{CI}}{\text{RI}}. \end{array}$$
In the formula, when CR < 0.1, there is good consistency.
This extension establishes the evaluation index set
The first-level evaluation index set is represented by *Z*, then
  (6) $$\begin{array}{c} Z=\left\{Z_{1},Z_{2},Z_{3,},\ldots ,Z_{n}\right\}. \end{array}$$
The corresponding weight set is represented by A, then
  (7) $$\begin{array}{c} A=\left\{a_{1},a_{2},a_{3},\ldots ,a_{n}\right\}. \end{array}$$
The secondary evaluation index set is represented by *Z*_*k*_, then
  (8) $$\begin{array}{c} Z_{k}=\left\{Z_{k1},Z_{k2},Z_{k3},\ldots ,Z_{\text{km}}\right\}. \end{array}$$
The corresponding weight set is represented by *A*_*k*_, then
  (9) $$\begin{array}{c} A_{k}=\left\{a_{k1},a_{k2},a_{k3},\ldots ,a_{\text{kn}}\right\}. \end{array}$$
The comment set is represented by W, then
  (10) $$\begin{array}{c} W=\left\{W_{1},W_{2},\ldots ,W_{L}\right\}. \end{array}$$
In this paper, *L* = 4, where the larger the *L* is, the smaller the score is, and the values are 100, 80, 60, and 40, namely
  (11) $$\begin{array}{c} W=\left(100,80,60,40\right). \end{array}$$
This leads to the evaluation matrix
  (12) $$\begin{array}{c} R_{k}=\left[\begin{array}{c} r_{11}r_{12}\cdots r_{1L}\\ r_{21}r_{22}\cdots r_{2L}\\ \cdots \\ r_{n1}r_{n2}\cdots r_{\text{nL}} \end{array}\right]. \end{array}$$
Thus, there are
  (13) $$\begin{array}{c} r_{\text{ij}}=\frac{W_{\text{ij}}}{\sum_{i=1}^{n}W_{\text{ij}}}. \end{array}$$
The evaluation matrix for this operation is obtained, and the subsidiary vector *B*_k_ of the secondary evaluation index *Z*_*k*_ to W is obtained as follows:
  (14) $$\begin{array}{c} B_{k}=A_{k}\times R_{k}. \end{array}$$
The vector set is represented by *R*, then
  (15) $$\begin{array}{c} R=\left[\begin{array}{c} B_{1}\\ B_{2}\\ .\\ B_{k} \end{array}\right]=\left[\begin{array}{c} b_{11}b_{12}\cdots b_{1L}\\ b_{21}b_{22}\cdots b_{2L}\\ \cdots \\ b_{n1}b_{n2}\cdots b_{\text{nL}} \end{array}\right]. \end{array}$$
Then use *R* to operate the evaluation matrix to obtain the auxiliary vector B of the first-level evaluation index *Z* to W
  (16) $$\begin{array}{c} B=A\times R=\left(b_{1},b_{2},\ldots ,b_{n}\right). \end{array}$$
When ∑_*j*=1_^*n*^*b*_*j*_ ≠ 1, normalize
  (17) $$\begin{array}{c} \tilde{b_{j}}=\frac{b_{j}}{\sum_{j=1}^{n}b_{j}},\\ \tilde{B}=\left(\tilde{b_{1}},\tilde{b_{2}},\ldots ,\overset{ˇ}{b_{n}}\right). \end{array}$$
Finally, a comprehensive evaluation model is obtained as follows:
  (18) $$\begin{array}{c} B=A\times R=A\times \left[\begin{array}{c} B_{1}\\ B_{2}\\ .\\ B_{k} \end{array}\right]=\left\{a_{1},a_{2},a_{3},\ldots ,a_{n}\right\}\times \left[\begin{array}{c} A_{1}\times R_{1}\\ A_{2}\times R_{2}\\ .\\ A_{n}\times R_{n} \end{array}\right]. \end{array}$$
(2) Construction of teaching system. In this paper, the physiology and medicine teaching system is divided into a common user module and an administrator module. The common user module includes several sections such as user login, course study, forum answering questions, and evaluation feedback. The course learning section includes several parts such as course search and course browsing and playback; the administrator module includes several major sections such as administrator login, course management, and website management. Course management also includes the release of course teaching videos, assignment of assignments, etc., as shown in Figure 7 [22].

Using the above system and the main content of the healthcare system builds a physiology and medicine teaching resource library and combines the human-computer interaction technology of the mobile app to build a modern healthcare system, as shown in Figure 8, in order to achieve the goal that everyone can study physiology and medicine teaching courses anytime and anywhere, thereby promoting national health care.

RETRACTED

### 4.2. System Testing and Evaluation

In order to understand the practical feasibility of this idea, this paper conducts a market test on the designed physiology and medicine teaching system, and the test environment is shown in Table 3.

The test method combined online questionnaires, in-app survey feedback, and field visits, and randomly selected 600 evaluation opinions. Statistical analysis was performed on this, and the results are shown in Figure 9.

It can be seen from Figure 9 that the evaluations of W1 (i.e., 80–100 points) and W2 (60–80 points) are significantly more than those of W3 (40–60 points) and W4 (below 40 points). A score above 60 is considered satisfactory, and the satisfaction of all aspects of the system can be shown in Figure 10.

It can be seen from Figure 10 that the user satisfaction with the overall content of the teaching system is as high as 86.33%, the user satisfaction with the convenience and performance of the system is as high as 95.17%, and the satisfaction with technical services is also 63.83%, with an average satisfaction of 81.78%. It can be said that the system meets the requirements of most people and can be loved by most people.

In addition, because ordinary users focus on performance, administrators pay more attention to management performance and efficiency. Based on the 600 questionnaires selected, this paper summarizes the use of the two on the teaching system, as shown in Table 4.

RETRACTED

The data show that in the 600 questionnaires selected, the evaluations of users and administrators are relatively satisfactory, and the administrators' evaluation of the teaching system is slightly lower than that of users. Few administrators are particularly satisfied with this system, and the majority are relatively satisfied, about 24% are dissatisfied, and only 15.7% are dissatisfied with this system, which shows that the system designed in this paper still has a lot of advantages room for improvement.

## 5. Discussion

In the design process of the system, this paper can realize the use of most functions to a certain extent. However, there are still some deficiencies in the beauty of the system interface, the convenience of the interactive interface, the integration of the database, the security of the data, and the running performance of the system. First, the quality of the website should be well reflected in its appearance. When the art and layout of the website are found to be not very good on the user side, users often unknowingly feel that other aspects of the website are not good enough. The most important part of a website's success is how it looks. The degree of aesthetics mentioned here does not mean how gorgeous the page is. Instead, lessons can be learned from traditional aesthetics; that is, the more beautiful something is, the more comfortable it will give. So, when designing a web page, we also need to put more effort into designing a beautiful, elegant, and unique page. In addition, many technologies need to be combined to achieve, and page layout and layout are also an issue worthy of our attention. No matter how perfect the style and aesthetics of the page are, there is no way to have a good page layout. Among them, the uniformity of page display needs to be realized in different browsers and different operating systems, which should also take into account the generality of HTML codes. When designing a page, read the HTML code carefully and make changes. We also need to learn a set of commonly used HTML coding standards [23].

Second, the system development process requires a very deep understanding of the basic principles and use of the database before proceeding with a rigorous database development program. We should also analyze the requirements of the database system, according to its functions after successful development and its subsequent data storage work. In the process of using the database, the SQL statement must also be mastered more completely. In addition, the adoption of technology in other databases is also critical. For example, the use of database views, stored procedures, and indexes is also essential [24].

RETRACTED

Finally, in addition to the above-mentioned problems, the operational performance and safety of the system must also be considered. In the process of program development, we need to pay more attention to the generality of the code, the balance of the code compilation system, and the database server, and consider the transmission speed of web page data from the server side to the browser side. From a security perspective, on the one hand, we also need to configure security settings based on user and privileged capabilities specific to your database system. On the other hand, we also need better control over the program code. For example, when logging in to the page, you can set irregular verification code input to prevent the possibility of brute force cracking.

## 6. Conclusions

This paper first gives a brief description of the overall content in the abstract part and then introduces the background significance and innovative points of this paper in the citation part and then cites some scholars' cases related to this research in the related work. Then, this paper analyzes the current situation of the domestic healthcare system, including the problems it faces. Next, this paper introduces the current situation of physiology and medicine teaching and the defects of traditional teaching methods, and proposes a teaching method combining the Internet and human-computer interaction. This paper introduces the concept, origin, and development of human-computer interaction in detail, and the design and classification of human-computer interaction, and proposes the basic content of the healthcare system based on human-computer interaction. Finally, it builds the teaching system evaluation model and the physiology and medicine teaching system framework, and shows the specific content of the modern health care system. In order to understand the practical feasibility of the system, this paper conducts market tests on the designed physiology and medicine teaching system. The test results show that the system has high practicability, can meet the needs of most users, and is more popular with most people. However, there are still areas where technical services are not perfect, and there is still room for development.

## Figures and Tables

**Figure 1:** 2016–2020 healthcare market. (a) Market size of medical devices. (b) Market scale of health checkup.

**Figure 2:** Traditional medical system.

**Figure 3:** Traditional physiology and medicine teaching.

**Figure 4:** Schematic diagram of human-computer interaction.

**Figure 5:** Interaction design principles. (a) Traditional interaction design principles. (b) Principles of modern interaction design.

**Figure 6:** Healthcare system.

RETRACTED

**Figure 7:** Framework of physiology and medicine teaching system.

**Figure 8:** Modern healthcare system.

**Figure 9:** System test feedback. (a) High evaluation feedback. (b) Low evaluation feedback.

**Figure 10:** Teaching system satisfaction.

**Table 1:** Status of domestic health and medical institutions.

Item	Number
Medical and health institutions	993 thousand
Health technician	8840 thousand
Total medical expenses: Yuan	3000 billion

**Table 2:** Physiological and medical teaching evaluation index assignment matrix.

Index	Content	Easy to use	Technical service	User satisfaction
Content	1	3	4	6
Easy to use	1/3	1	2	4
Technical service	1/4	1/2	1	3
User satisfaction	1/6	1/4	1/3	1

**Table 3:** Teaching system test environment.

Class	Content
Test object	User, administrator
Test the network environment	4 G, 5 G, Wi-Fi
Test port	Android, iPhones, iPad, tablet

**Table 4:** System satisfaction survey statistics.

Evaluation	User	Administrator
Number	437	163
Extremely dissatisfied	1	3
Dissatisfied	69	36
Relatively satisfied	212	104
Very satisfied	155	20

## Data Availability

The data that support the findings of this study are available from the corresponding author upon reasonable request.
